This article has been retracted.

# Muscone Inhibits the Excessive Inflammatory Response in Myocardial Infarction by Targeting TREM-1

**DOI:** 10.1155/2022/9112479

**Published:** 2022-05-10

**Authors:** Hong Zhang, Jian Ye, Xu Wang, Zongjun Liu, Tao Chen, Junqing Gao

**Affiliations:** Department of Cardiology, Putuo Hospital, Shanghai University of Traditional Chinese Medicine, Shanghai 200062, China

## Abstract

The inhibitory effect of muscone on the hyperinflammatory response after myocardial ischemia reperfusion injury (MIRI) was investigated, and the target and signal pathways of muscone were explored. The levels of inflammatory cytokines interleukin-1*β*, interleukin-6, and tumor necrosis factor alpha were detected through qRT-PCR and ELISA. The expression levels of p38 and NF-*κ*B signaling pathway-related proteins were detected through Western blot. TREM-1 siRNA was transfected into macrophages in vitro. The rat model of myocardial ischemia was established and used in studying the inhibitory effect of muscone on the inflammatory response and its protective effect muscone on myocardial apoptosis. The expression of TREM-1 was upregulated during myocardial ischemia. Knocking down TREM-1 decreased the increase in inflammatory cytokines in the supernatant of macrophages induced by rmHMGB1 (1 *μ*g/mL) and rmHSP60 (1 mol/mL). In addition, knocking down TREM-1 decreased p38 and NF-*κ*B signaling activation. Muscone can protect myocardial cells by inhibiting the expression of TREM-1 and the inflammatory response after myocardial infarction. Further study showed that muscone inhibited the production of DAM-triggered (damage-associated molecular pattern trigger) inflammatory cytokines. In addition, muscone inhibited the activation of p38 and NF-*κ*B signals under DAM-induced conditions. Muscone and TREM-1 gene knockout reduced cell apoptosis and provided protection against MIRI by inhibiting p38 and NF-*κ*B signaling activation. Mechanism studies showed that muscone inhibited the production and release of inflammatory cytokines by inhibiting TREM-1, and thereby reducing the inflammatory response and providing protection against MIRI.

## 1. Introduction

Myocardial ischemia reperfusion injury (MIRI) is a complex pathophysiological process with multiple factors and pathways [1], but the mechanism of MIRI has not been fully elucidated [2]. Free radical burst, calcium overload, myocardial energy metabolism disorder, endothelial cell dysfunction, neutrophil infiltration, apoptosis, and mitochondrial damage during myocardial reperfusion are considered important factors for the occurrence and development of MIRI [3]. Thus, determining how to reduce MIRI is particularly important. Apoptosis is one of the important mechanisms of myocardial cell death in acute MIRI [4], and the inflammatory response is an important mechanism causing MIRI [5].

Triggering receptors expressed on myeloid cells (TREMs) constitute a family of triggering receptors expressed on the surfaces of neutrophils and monocytes [6]. These receptors can induce the expression of inflammatory cytokines and adhesion molecules and promote the mature immune regulation of dendritic cells [7]. TREMs play an important role in the inflammatory response. TREM-1 is a novel inflammation-triggering receptor, which plays an important role in intrinsic immunity against severe infection and sepsis [8]. TREM-1 amplifies inflammation and is a major mediator of inflammation [9]. In experimental animals with lipopolysaccharide (LPS)-induced septic shock, overreaction and death are prevented by blocking the TREM-1 signaling.

Muscone (3-methylcyclopentadecanone) is the main active ingredient in artificial musk and has antidementia, anticerebral ischemia, anti-inflammation, and other pharmacological effects [10–12]. It can reduce secondary injuries, such as edema, inflammation, neuron degeneration, and necrosis after spinal cord injury and promote nerve recovery in rats [13]. Moreover, it can provide protection against acute cerebral ischemia injury [14, 15]. However, whether muscone can improve myocardial ischemia by inhibiting TREM-1 is unclear.

The purpose of this study was to observe the protective effect of muscone against acute MIRI in rats and study the effect of muscone on the TREM-1 pathway. In addition, the anti-inflammatory mechanism of muscone in the treatment of MIRI was studied. This study provides insights into and experimental basis for the clinical application of muscone in the prevention and treatment of coronary heart diseases.

## 2. Materials and Methods

### 2.1. Animal Model of Myocardial Ischemia

SPF healthy adult Sprague–Dawley rats (males, body weights of 200–240 g, aged 7 weeks) were purchased from Sipeifu (Beijing) Biotechnology Co., Ltd. The rats were divided into the sham, MIRI model, and MIRI + muscone groups. Each group contained six rats. Muscone was purchased from Aladdin (541-91-3, purity of >97%, Beijing, China). Muscone was dissolved in normal saline. For the MI model, the dose of muscone was 2 mg/kg/day, and the treatment was performed through intragastric administration [16]. The rats were intraperitoneally anesthetized with pentobarbital sodium (50 mg/kg). The trachea was intubated and fixed in an inverted position. Artificial respiration was performed by connecting a small animal ventilator and an ECG machine. Thoracotomy was performed, three or four ribs were broken, and the pericardium was opened to expose the heart. The left anterior descending coronary artery was threaded approximately 2 mm below the bifurcation with a No. 0 surgical thread. The drug or saline was administered to the tail vein. After stabilization for 10 min, ligation was performed, and the chest was closed. Increased QRS amplitude, ST segment elevation, *T* wave elevation, or inversion was used as the criterion for determining the success of ischemia. The reperfusion injury process was achieved by cutting a ligation line 35 min after ligation. The chest wall was sutured, and the animal resumed breathing on its own. Approximately 150 min after reperfusion, the rats were intraperitoneally anesthetized with pentobarbital sodium. Blood and cardiac tissue samples were collected for testing. The sham operation group was only threaded without ligation, and the other operations were the same as those used in the model group. The desired concentrations of the drug were prepared with saline. Immediately after the threading of the left anterior descending coronary artery, the drug was injected into the caudal vein once. The sham operation and model groups received normal saline. This study was approved by the ethics committee of Putuo Hospital.

### 2.2. Pathological Changes in Myocardial Tissues Were Observed through HE Staining

The myocardial tissue was removed after reperfusion. After rinsing with phosphate buffer solution (PBS), the samples were fixed with 4% paraformaldehyde at 4°C for 24 h, washed with PBS three times, and dehydrated with 30%, 50%, and 70% alcohol successively for 10 min for each concentration. Then, the samples were dehydrated in a dehydrator and embedded in paraffin before sectioning. Finally, staining was performed according to the operation instructions provided by the HE staining solution kit. Pathological changes in the myocardial tissues were observed under a microscope.

### 2.3. Cell Culture

RAW264.7 cells were purchased from American Type Culture Collection (ATCC, Manassas, VA, USA) and inoculated in a PRIM1640 medium containing 10% fetal bovine serum (Gibco, Life Technologies, Rockville, MD, USA). The cells were cultured at 37°C in a 5% CO_2_ incubator. The cells were inoculated into Petri dishes. After 24 h of culture, the medium was replaced with a serum-free medium, and the cells were cultured overnight. Recombinant mouse HMGB1 (rmHMGB1; ab255799 Abcam, Cambridge, MA, USA) and recombinant mouse Hsp60 (rmHSP60; ab92364) were purchased from Abcam. rmHMGB1 (1 *μ*g/mL) and rmHSP60 (1 mol/mL, 6 h) were used in constructing an induction model [17]. Drugs were added 1 h before the model construction. Total protein or total RNA was extracted at different time points according to experiment requirements.

### 2.4. Cell Transfection

Macrophages were cultured in vitro. The macrophages in the exponential growth phase were removed from the incubator and observed under a microscope. TREM-1 siRNA (sc-43000, Santa Cruz Biotechnology, Dallas, TX, United States) was transfected into the macrophages with Lipofectamine 2000 (Life Technologies, Rockville, MD, USA). The target sequence used for TREM-1 was 5′-CACGTATCTTATCAGGAAA-3′ (50 *μ*g). The silencing effect of TREM-1 was verified with qRT-PCR 24 h later.

### 2.5. Quantitative PCR

The TRIzol reagent was used in extracting total RNA from the cultured cells. cDNA was synthesized with a reverse transcription reaction system and 1 *μ*g of total RNA. This method was used as the template PCR method for amplification. The primers used in the PCR reaction were as follows: TREM-1, forward primer, 5′-TATGCCAACAGCCAGAAGGC-3′; TREM-1, reverse primer, 5′-GGGTTCCTTCCCGTCTGGTA-3′; interleukin-1*β* (IL-1*β*; upstream), 5′-TGAAGGGCTGCTTCCAAACCTTTGACC-3′; IL-1*β* (downstream), 5′-TGTCCATTGAGGTGGAGAGCTTTCAGC-3′; interleukin-6 (IL-6; upstream), 5′-TGAACAACGATGATGCACTTGC-3′; IL-6 (downstream), 5′-CGTAGAGAACAACATAAGTC-3′; tumor necrosis factor alpha (TNF-*α*; upstream), 5′-CCCTCACACTCAGATCATCTTCTCAA-3′; TNF-*α* (downstream), 5′-GAATTCGGAAAGCCCATTTGAGTCC-3′; GAPDH (upstream), 5′-AAGTTCAACGGCACAGTCAA-3′; upstream, 5′-TACTCAGCACCAGCATCACC-3′ Mix SYBR (5 *μ*L); upstream and downstream primers (0.3 *μ*L each); DEPC water (3.4 *μ*L); and cDNA (1 *μ*L). The reaction conditions were as follows: 94°C for 2 min, 92°C for 20 s, 56°C for 30 s, and 72°C for 45 s (total of 30 cycles). The last PCR extension was performed at 72°C for 7 min. The relative expression of each gene was calculated with the 2^-△△^CT method.

### 2.6. Western Blot

Protein lysis and protein quantification were performed with the BCA method. A protein loading buffer (5×) was added and placed in boiling water for 10 min for the complete denaturation of the protein. After SDS-PAGE separation, the protein was transferred to a PVDF membrane. BSA (5%) was sealed for 1 h. A diluted primary antibody was added. P38 (1 : 1000, ab170099, Abcam, Cambridge, MA, USA), p-p38 (ab178867), JNK (ab199380), p-JNK (ab124956), p65 (ab32536), p-p65 (ab183559), and GAPDH (ab181602) were added. The membrane was incubated overnight in a refrigerator at 4°C, and then was washed with TBST five times, and incubated with a horseradish peroxidase labeled secondary antibody (1 : 1000, ab7090 and ab7069) at room temperature for 2 h. The membrane was washed with TBST five times, and the enhanced chemiluminescent reagent was added for the quantification of protein expression. Grayscale analysis was performed with a system imaging software. The protein expression level was indicated by the ratio of protein expression in myocardium tissues of each group to that of the internal reference GAPDH. The gray values of the protein bands were determined using Image *J* (V1.8.0.112).

### 2.7. ELISA

RAT IL-6 ELISA kit (RayBio, Lot#1229170724) and RAT IL-1 Beta ELISA kit (RayBio, Lot#1229170721) were used. After the modeling, blood was collected from the abdominal aorta. The serum was separated through centrifugation at 3000 g/min for 10 min after standing at room temperature for 1 h in a natural state. The levels of TNF-*α*, IL-6, and IL-1*β* were determined according to the kit instructions. Serum CK, AST, and LDH activities were measured with a COBAS-FARA automatic biochemical analyzer (Roche, Basel, Switzerland).

### 2.8. TUNEL Staining

The paraffin sections of the prepared cardiac tissues were placed in an oven at 60°C and baked for 2 h. After 20 *μ*g/mL proteinase K was added, the sections were incubated at room temperature for 15 min. After rinsing with PBS, 50 *μ*L of TUNEL assay solution (Beyotime, Shanghai, China) was added to the sections, which were incubated at 37°C for 1 h. The paraffin sections were stained with fluorescence dyes and observed under a fluorescence microscope (Nikon, Japan). Apoptotic cells were counted using Image-Pro Plus 6.0 image analysis software. The apoptosis rates of the cardiomyocytes were determined using the formula apoptotic index = number of apoptotic cardiomyocytes/the total number of cardiomyocytes × 100.

### 2.9. Statistical Analysis

SPSS 20.0 (SPSS Inc., Chicago, IL, USA) was used. The measurement data obtained from the experiment were expressed as mean ± standard deviation. One-way analysis of variance was used in comparing multiple groups, and the Tukey test was used for determining the homogeneity of variance. Unpaired Student's *t*-test was used in comparing two groups. A *P* value of <0.05 indicated a statistically significant difference.

## 3. Results

### 3.1. Expression of TREM-1 was Upregulated after Myocardial Infarction

To study the role of TREM-1 in myocardial infarction and inflammation, we constructed an animal model of MIRI. The results of HE staining showed that the myocardial tissue of the sham operation group was orderly and showed no degeneration. Cell necrosis was observed, but no inflammation occurred in the interstitium. In the model group, the myocardial tissue was disordered, and edema and cardiomyocyte degeneration, interstitial edema, and vascular hyperplasia and dilation occurred (Figure 1(a)). Subsequently, the mRNA levels of IL-1*β*, IL-6, and TNF*α* were detected in the myocardial tissues through qRT-PCR. The expression levels of IL-1*β*, IL-6, and TNF*α* were upregulated in the myocardial tissues of rats in the model group (Figure 1(b)–1(d)) compared with those in the sham operation group. Compared with the sham operation group, the expression of Bax in the myocardial tissue of the MI model group was also upregulated (Figure 1(e)). The Bcl-2 expression was downregulated (Figure 1(f)). qRT-PCR results showed that the expression of TREM-1 in the myocardial tissues of rats in the model group was upregulated (Figure 1(g)) compared with that in the sham operation group. The expression levels of HMGB1 and HSP60 in the heart tissue homogenates of rats in the myocardial infarction model group or those subjected to sham operation were determined by ELISA. The expression levels were upregulated after myocardial ischemia (Figure 1(h)–1(i)). Furthermore, Western blot was used in detecting the expression levels of HMGB1 and HSP60 in the heart tissue homogenates of rats in the myocardial infarction model group or those subjected to sham operation. HMGB1 and HSP60 expression levels were upregulated after myocardial ischemia (Figure 1(j)).

### 3.2. Knocking Down TREM-1 Reduced the Production of Inflammatory Cytokines Induced by DAM-Induced Inflammation

The results of the investigation on the high knockdown efficiency of siRNA TREM-1 showed that siRNA can effectively reduce the TREM-1 expression (Figure 2(a)). Knocking down TREM-1 inhibited the increase in inflammatory cytokines in the macrophage supernatant induced by rmHMGB1 (1 *μ*g/mL). After knocking down TREM-1, IL-1*β*, IL-6, and TNF*α* levels in the macrophages decreased (Figure 2(b)). In addition, TREM-1 knockdown inhibited the increase in inflammatory cytokines in the macrophage supernatant induced by rmHSP60 (1 mol/mL). After TREM-1 was knocked down, IL-1*β*, IL-6, and TNF*α* levels in the macrophages decreased (Figure 2(c)).

### 3.3. Knocking Down TREM-1 Reduced the Signal Activation of P38 and NF-*κ*B under a DAM-Induced Condition

The expression level of p-p38 in macrophages in the rmHMGB1- and rmHSP60-induced groups significantly increased compared with that in the control (CTRL) group. The expression level of p-p38 decreased after TREM-1 knockdown compared with that in the induction group. The Western blot results showed that the expression levels of p-JNK and p-p65 increased after the induction of rmHMGB1 and rmHSP60. However, the expression of p-JNK and p-p65 decreased after TREM-1 knockdown. TREM-1 knockdown inhibited the signal activation of p38 and NF-*κ*B under a DAM-induced condition (Figure 3(a)–3(b)).

### 3.4. Muscone Inhibited the Inflammatory Response after Myocardial Infarction and Protected Myocardial Cells

We investigated the role of muscone in myocardial infarction and inflammation in the animal models of MIRI.  Figure 4(a) shows the molecular structure of muscone. The results of HE staining showed that the myocardial tissue of the MI model was disordered and presented edema, cardiomyocyte degeneration, interstitial edema, vascular hyperplasia and dilation. However, muscone treatment resulted in the orderly arrangement of myocardial tissues and reduced necrosis and inflammatory cell infiltration (Figure 4(b)). Muscone treatment prevented edema, cardiomyocyte degeneration, vascular hyperplasia and dilation induced by MIRI. We used qRT-PCR to detect the mRNA levels of IL-1*β*, IL-6, and TNF*α* in the myocardial tissues. The expression levels of IL-1*β*, IL-6, and TNF*α* in the myocardium of the model group were upregulated compared with those in the sham operation group. The expression levels of IL-1*β*, IL-6, and TNF*α* in the myocardial group decreased after muscone treatment (Figure 4(c)–4(e)) compared with those in the model group. We used ELISA to detect the serum levels of AST, CK, and LDH. The serum levels in the model group were upregulated compared with those in the sham operation group. The serum level decreased after muscone treatment (Figure 4(f)–4(h)) compared with that in the model group. These results showed that muscone treatment reduced serum myocardial injury markers. To analyze the effect of muscone on apoptosis in rats with MIRI, we used TUNEL to detect cell apoptosis. The TUNEL staining results of the myocardial tissues showed that the apoptotic cells increased in the MIRI group compared with those in the CTRL group. Compared with the apoptosis cells in the MIRI group, the apoptosis cells in the myocardial tissues in the MIRI + muscone group decreased (Figure 4(i)). The expression level of Bax increased, whereas that of Bcl-2 decreased in the MIRI group, relative to those in the CTRL group. Compared with the MIRI group, the expression of Bax decreased and the expression of Bcl-2 increased in the myocardial tissues of rats in the MIRI + muscone group (Figure 4(j)–4(k)). The qRT-PCR results showed that muscone inhibited the expression of TREM-1 (Figure 4(l)). In conclusion, muscone can reduce cell apoptosis in rats with MIRI by inhibiting TREM-1 expression.

### 3.5. Targeted Inhibition of TREM-1 by Muscone

In the macrophages, rmHMGB1 induction stimulated the upregulation of TREM-1 expression (Figure 5(a)). Muscone treatment decreased the expression of TREM-1 (Figure 5(b)). In the macrophages, rmHSP60 induction upregulated the expression of TREM-1 (Figure 5(c)). Muscone inhibited the upregulation of TREM-1 expression induced by rmHSP60 (Figure 5(d)).

### 3.6. Muscone Inhibited the Production of Inflammatory Cytokines and Inhibited the Signaling Activation of p38 and NF-*κ*B

Figure 6(a) shows that muscone inhibited the increase in inflammatory cytokines in the supernatant of macrophages induced by rmHMGB1 (1 *μ*g/mL). The levels of IL-1*β*, IL-6, and TNF*α* in the macrophages decreased after muscone treatment. Muscone inhibited the increase in inflammatory cytokines in the supernatant of macrophages induced by rmHSP60 (1 mol/mL). After muscone treatment, the levels of IL-1*β*, IL-6, and TNF*α* in the macrophages decreased (Figure 6(b)). The effects of muscone on p38 and NF-*κ*B signaling pathways in rats with MIRI were analyzed by detecting the protein expression levels of the p38 and NF-*κ*B signaling pathways. The Western blot results showed that the expression levels of p-p38, p-JNK, and p-p65 were upregulated after rmHMGB1 and rmHSP60 induction, relative to those in the CTRL group. By contrast, the expression levels of p-p38, p-JNK, and p-p65 decreased after muscone treatment (Figure 6(c)–6(d)).

## 4. Discussion

Inflammation is the key pathological mechanism of MIRI [18]. During myocardial ischemia, the apoptosis rates of the cardiomyocytes increases, and reperfusion aggravates inflammatory response; various inflammatory factors are involved in MIRI and aggravate myocardial injury [19]. Many traditional Chinese medicine extracts can regulate cell apoptosis, oxidative stress, and inflammation, playing a positive role in the treatment of various diseases. Liu et al. [20] found that shionin can reduce edema and necrosis of liver tissues, reduce AST and ALT levels, reduce Bax expression, and increase the Bcl-2 expression in rats with acute liver injury induced by concanavalin A.

TREM-1 is an important member of the TREM family, specifically belonging to a family of receptors associated with NK cell receptors. TREM-1 can activate downstream signaling events with the help of a junction protein named DAP12 [21–23]. The expression of TREM-1 in cells was induced by LPSs and lipoteichoic acid, ligands of TLR4. Although the ligand of TREM-1 is unknown, the binding of TREM-1 on monocytes to anti-MABs causes the production of proinflammatory cytokines, such as TNF-*α* and IL-1*β*, and cytokines such as interleukin-8 and monocyte chemotactic protein 1. The binding of TREM-1 to a bacterial ligand activating Toll-like receptors synergically increases the production of proinflammatory cytokines TNF-*α* and granulocyte-macrophage stimulating factor while inhibiting the production of anti-inflammatory cytokine interleukin-10. The results of this study showed that TREM-1 expression was up-regulated in MIRI. TREM-1 knockdown reduces the levels of inflammatory cytokines, HMGB1- and HSP60-induced inflammatory responses, and p38, p-JNK, and p-p65 protein levels.

Muscone has an antimyocardial ischemia effect. The experimental animal model of myocardial ischemia in rats showed that muscone inhibited myocardial ischemia by exerting an antihypoxic effect, reducing the *T* peak of ECG and CK and LDH [10–12]. Muscone suppresses the inflammatory response. Liang et al. [24] found that muscone (10 mg/kg) can significantly downregulate the expression levels of TNF-*α*, IL-1*β*, PGE2, 6-ketoprostatin F, and other inflammatory cytokines in rats. In vitro experiments showed that muscone can inhibit the production of TNF-*α*, IL-1*β*, cyclooxygenase-2, nitric oxide, inhibitory nitric oxide synthase, and MMP-13. In this study, we found that the serum TNF-*α*, IL-6, and IL-1*β* levels of animals treated with muscone significantly decreased compared with those in the ischemia-reperfusion group. These results indicated that muscone can reduce the inflammatory response by inhibiting the production of TNF-*α*, IL-6, and IL-1*β* and reduces the inflammatory damage caused by it. Therefore, the inhibition of TREM-1 and inflammatory response may be one of the mechanisms by which muscone protects the myocardium against ischemia reperfusion injury. The results of this study showed that muscone can reduce the levels of myocardial injury markers and inflammatory factors and reduce cell apoptosis in rats with MIRI. The mechanism studies showed that muscone inhibited the expression of TREM-1, decreased the expression of Bax, and enhanced the expression of Bcl-2.

Muscone exerted a significant inhibitory effect on MIRI in the animal and cell experiments. The results of the present study showed TREM-1 is a potential target protein. However, whether other targets need to be further studied is unclear. In addition, the downstream mechanisms of TREM-1 were implicated in this study.

## 5. Conclusion

Muscone can protect myocardial tissues and reduce myocardial cell apoptosis and injury.

Muscone can reduce TNF-*α*, IL-6, and IL-1*β* levels in myocardial tissues. In addition, muscone can reduce serum AST, CK, and LDH levels. The mechanism may involve the inhibition of TREM-1, subsequent inhibition of NF-*κ*B, inhibited production of TNF-*α*, IL-6, and other inflammatory factors. This mechanism protects the myocardium.

## Figures and Tables

**Figure 1:** Inflammation and apoptosis are increased during myocardial ischemia-reperfusion injury and the TREM-1 expression was upregulated after myocardial infarction. (a). HE staining confirms the successful modeling of myocardial ischemia. (b). qRT-PCR detects the mRNA expression of IL-1*β* in the myocardial tissue of the sham group and MI model. (c). qRT-PCR detects the mRNA expression of IL-6 in the myocardial tissue of the sham group and MI model. (d). qRT-PCR detects the mRNA expression of TNF*α*in the myocardial tissue of the sham group and MI model. (e). qRT-PCR detects the mRNA expression of Bax in the myocardial tissue of the sham group and MI model. (f). qRT-PCR detection of the Bcl-2 mRNA expression in the myocardial tissue of the sham group and MI model. (g). qRT-PCR detection of the TREM-1 mRNA expression in the myocardial tissue of the sham group and MI model. The TREM-1 expression is upregulated during myocardial ischemia. (h). ELISA was used to detect the content of HMGB1 in rat heart tissue homogenate after myocardial infarction model group or sham operation. (I) ELISA was used to detect the production of HSP60 in rat heart tissue homogenate after myocardial infarction model group or sham operation. (J) Western blot was used to detect the production of HMGB1 and HSP60 in rat heart tissue homogenate after myocardial infarction model group or sham operation. ^*∗∗*^*P* < 0.01.

**Figure 2:** Knockdown of TREM-1 reduces the production of inflammatory cytokines triggered by DAMP-induced. (a). Verification of siRNA TREM-1 knockdown efficiency. QRT-PCR detection of TREM-1 mRNA expression in si-NC and si-TERM-1 group. (b). Knockdown of TREM-1 reduces rmHMGB1 (1 *μ*g/ml) induced an increase in cytoinflammatory factors in the supernatant of macrophages. (c). Knockdown of TREM-1 reduces rmHSP60 (1 mol/ml) induced an increase cytoinflammatory factors in the supernatant of macrophages. ^*∗∗*^*P* < 0.01.

**Figure 3:** Knockdown of TREM-1 reduces the signal activation of p38 and NF-*κ*B under DAMP-induced conditions. (a). Western blot detects the changes in p-p38 and p-p65 and p-JNK expression in each group after different treatments. (b). Statistical results of p-p38 and p-p65 and p-JNK expression. ^*∗∗*^*P* < 0.01.

**Figure 4:** Muscone inhibits inflammation and apoptosis after myocardial infarction and protects myocardial cells. (a). The molecular structure of Muscone. (b). HE staining results of the myocardial tissue in different treatment groups. (c). qRT-PCR detects the mRNA expression of IL-1*β* in the myocardial tissue of different treatment groups. (d). qRT-PCR detects the mRNA expression of IL-6 in the myocardial tissue. (e). qRT-PCR detects the mRNA expression of TNF*α* in myocardial tissues. (f). ELISA detects the content of AST in in the serum of different treatment groups. (g). ELISA detects the content of CK in in serum of different treatment groups. (h). ELISA detects the content of LDH in the serum of different treatment groups. (i). Myocardial tissue TUNEL detects the degree of apoptosis. (j). qRT-PCR detects the mRNA expression of Bax in myocardial tissues. (k). qRT-PCR detection of the Bcl-2 mRNA expression in myocardial tissues. (l). Muscone inhibits the expression of TREM-1. ^*∗∗*^*P* < 0.01.

**Figure 5:** Muscone targets TREM-1 and inhibits its expression. (a). In macrophages, rmHMGB1 induces an upregulation of the TREM-1 expression. (b). In macrophages, muscone inhibits the upregulation of the TREM-1 expression induced by rmHMGB1. (c). In macrophages, rmHSP60 induces an upregulation of the TREM-1 expression. (d). In macrophages, muscone inhibits the upregulation of the TREM-1 expression induced by rmHSP60. ^*∗∗*^*P* < 0.01.

**Figure 6:** Muscone inhibits the production of DAMP-triggered (damage-associated molecular pattern trigger) inflammatory cytokines. In addition, muscone inhibits the signal activation of p38 and NF-*κ*B under DAMP-induced conditions (a). Muscone inhibits rmHMGB1 (1 *μ*g/ml)-induced increase in cytoinflammatory factors in the supernatant of macrophages. (b). Muscone inhibits rmHSP60 (1 mol/ml)-induced increase in cytoinflammatory factors in the supernatant of macrophages. (c). Western blot was used to detect the expression in the p-p38, p-p65 and p-JNK expression in each group after different treatments. (d). Statistical results of p-p38, p-p65 and p-JNK expressions in each group after different treatments. ^*∗∗*^*P* < 0.01.

## Data Availability

The datasets used and/or analyzed during the current study are available from the corresponding author on reasonable request.
